The article "Improving measles vaccine uptake rates in Nigeria: An RCT evaluating the impact of incentive sizes and reminder calls on vaccine uptake" was retracted in 2020. Reasons: lack of ethics approval or compliance; concerns about the data; concerns about the authorship.

# Improving measles vaccine uptake rates in Nigeria: An RCT evaluating the impact of incentive sizes and reminder calls on vaccine uptake

**DOI:** 10.1371/journal.pone.0233149

**Published:** 2020-06-18

**Authors:** Steven Brownstone, Alison Connor, Daniel Stein

**Affiliations:** IDinsight, San Francisco, California, United States of America; IAVI, UNITED STATES

## Abstract

**Objective:**

To assess the impact of increasing incentive size and reminder calls on the measles vaccine uptake rate.

**Design:**

Randomized controlled trial, randomized at individual level, stratified by clinic.

**Setting:**

Nigeria

**Participants:**

1088 caregivers with children aged nine months or older; had received at least one previous conditional cash transfer (CCT) at a program clinic, had received their Penta-3 immunization but had not yet received their measles immunization, and the caregiver had provided a phone number.

**Intervention:**

Nine clinics were randomized to two models; caregivers in Model 1 received a default of 2000 Nigerian Naira (NGN) for completing the measles vaccine, and those in Model 2 received by 3000 NGN. Caregivers from the respective clinics were then randomized to one of the four arms: 1) control (baseline amount of 2000 NGN or 3000 NGN), 2) baseline amount plus a reminder call, 3) baseline amount plus 1000 NGN and a reminder call, and 4) baseline amount plus 3000 NGN and a reminder call.

**Main outcome measure:**

Receipt of measles vaccine as reported on a child health card.

**Results:**

Overall, there was no clear trend that increasing the incentive amount resulted in an increase in vaccine uptake rates. In Model 1 households, an additional 1000 NGN and 3000 NGN resulted in a 6.4 percentage point (95% CI: -2.3–15, p-value = 0.15) and 11.8 percentage point (95% CI: 3.9–19.6, p-value = 0.003) increase in the probability of completing the measles vaccines, respectively. This increase, however, was only significant for the 3000 NGN increase. On the other hand, in Model 2 households, increasing the incentive by 1000 NGN and 3000 NGN increased the probability by 3.3 (95% CI: -3.8–10.4, p-value = 0.36) and 3.3 (95% CI: -3.7–10.4, p-value = 0.35) percentage points. These increases were not statistically significant.

Adding reminder calls to CCTs increased the probability of completing the measles vaccine; caregivers who received reminder calls plus CCTs were 5.1 percentage points more likely to get their children vaccinated (95% CI: 0.50–9.8, p-value = 0.03) compared to those who received CCTs and did not receive a reminder call. These results were largely driven by caregivers who went to clinics in Model 1.

**Conclusion:**

A combination of increasing incentive amounts and reminder calls modestly improves measles immunization rates. However, this program also shows that there is substantial regional heterogeneity in response to both incentives and calls. While one possible conclusion is that a larger incentive and phone reminders are more likely to work in higher income and higher baseline coverage settings, the study is not designed to evaluate this claim. Rather, policymakers could consider experimenting with a similar low-cost calling study as part of the design of other cash transfer programs to identify whether adding reminder phone calls could increase the impact of the program.

## Introduction

Over the past decade, greater access to immunizations has led to fewer child deaths around the world [1]. Yet, vaccine-preventable diseases are still one of the major causes of death among children under the age of five in Sub-Saharan Africa [2]. Nigeria has the highest number of unimmunized children worldwide and is among the top 10 countries with incomplete immunizations [3].

In Nigeria, a child is considered to be fully vaccinated if he or she has received: a) a BCG immunization against tuberculosis and a Hepatitis B vaccine (at birth or as soon as possible after birth); b) three doses of PENTA to prevent diphtheria, pertussis (whooping cough), tetanus, Hepatitis B, and Haemophilus influenza type B (at 6, 10, and 14 weeks of age); c) at least three doses of oral polio vaccine (at 6, 10, and 14 weeks of age); and d) one dose of measles and yellow fever vaccines (at 9 months of age) [4].

The measles vaccine is considered one of the most important because measles has frequent breakouts, is highly contagious, and has a high mortality rate [1]. In Nigeria, measles vaccine coverage is at 42% compared to 72% across Sub-Saharan Africa [5] and 85% worldwide [1]. Coverage is particularly low in Northern Nigeria, with coverage estimates ranging from 22%-40% compared to 70%-73% in the South [5]. Recent research suggests the regional difference is more likely primarily driven by demand-side issues rather than supply-side factors.[6] Demand side factors include lack of knowledge, e.g., the importance of immunizations and their respective schedules, and myths and rumors about routine immunization [7,8].

New Incentives and the All Babies are Equal Initiative (NI-ABAE), non-profit organizations operating in North West Nigeria, implemented a conditional cash transfer (CCT) program to improve immunization coverage. It offered caregivers cash payments when they brought their children for immunization. They implemented two models with different incentive amounts in order to determine the optimal incentive amount that would increase immunization uptake rates. In Model 1, caregivers received 500 NGN (~1.39 USD) and in Model 2, caregivers received 1000 NGN (~2.78 USD) for each of the first four routine immunizations. For the measles vaccine, caregivers in Model 1 received 2000 NGN (~5.56 USD) while caregivers in Model 2 received 3000 NGN (~8.34 USD) (Table 1). This amount was intended to be sufficient to cover the caregiver’s transportation costs to the nearest health facility and also provide a small incentive for the mothers. All caregivers with listed numbers received SMS reminders prior to immunization due dates. For the purpose of this study, a proportion of caregivers were also given phone call reminders to remind them of their child’s immunization due date. This study sought to assess the impact of increasing cash incentives and reminder calls on measles immunization rates.

**Table 1:** NI-ABAE’s pay-out schedule.

Vaccine^§^	Timing	Payment amount (NGN)
BCG vaccine	Birth	500 (Model 1 clinics) 1000 (Model 2 clinics)
Pentavalent vaccine and PCV, dose 1	6 weeks	500 (Model 1 clinics) 1000 (Model 2 clinics)
Pentavalent vaccine and PCV, dose 2	10 weeks	500 (Model 1 clinics) 1000 (Model 2 clinics)
Pentavalent vaccine and PCV, dose 3	14 weeks	500 (Model 1 clinics) 1000 (Model 2 clinics)
Measles vaccine	9 months	2000 (Model 1 clinics) 3000 (Model 2 clinics)

^*§*^This list contains the immunizations listed in the eligibility criteria and not all the immunizations on the immunization schedule

The NI-ABAE’s intervention was based on the growing body of literature which suggests that non-monetary and monetary incentives can be effective in encouraging caregivers to immunize their children. In a randomized controlled trial (RCT) conducted in India, results showed a 30-percentage point increase in immunization rates in the incentivized arm compared to the arm that only received access to reliable immunization. Households were offered 1 kg of lentils (~$1) per immunization and *thalis* (dishes)(~$2) after the full course. [9] Similarly, in Pakistan, food or medicine vouchers worth $2 doubled the odds of completing the DPT vaccine series at 18 weeks of age [10]. Studies in Nicaragua and Honduras have also shown some increase in clinic attendance and immunization rates when families were offered food and cash [11,12].

Researchers have also explored the impact of incentive sizes on immunization rates and found mixed results. A cluster RCT conducted in Kenya revealed that children in the highest incentive group (SMS plus 200 Kenyan Shillings, KES) (~1.97 USD) were significantly more likely to achieve full immunization compared to the other groups (control, SMS only, and SMS plus 75 KES) [13]. Conversely, in the Banerjee et al. study, the highest incentive group achieved increases in immunization rates similar to those who received the lower incentive (2010). Banerjee et al. posit that the incentive size may not matter as much as the fact that there is an incentive in the first place (2010). This finding supports results from a study conducted in Cambodia that looked at the impact of cash incentives on school attendance which also suggested that a larger incentive may not necessarily increase outcomes [14].

Furthermore, researchers have explored the impact of reminders on immunization schedule completion [2,13,15]. In Zimbabwe, Bangure et al. found that immunization rates were higher for the people who received text message reminders; immunization coverage at six weeks after birth was 97% for those who received reminders and 82% for those who did not (p < 0.01), similarly at 14 weeks, immunization coverage was 95% for the intervention group and 75% for the control group (p < 0.01) (2015). This study also revealed that text message reminders improved immunization timeliness, that is, immunization within two weeks of the due date. At six weeks after birth, 93% of the mothers who received messages took their children for immunization within two weeks of the due date compared to 24% of mothers who did not receive messages (p<0.01). In addition to these studies, one study examined the effects of providing both incentives and text message reminders, revealing that this combination significantly increases the likelihood of immunization [13].

In 2017, IDinsight conducted an RCT to assess two components of NI-ABAE’s program: 1) Does increasing cash incentive amounts increase uptake of the measles vaccine among caregivers who are already enrolled in their program? 2) Does giving phone reminders to caregivers who are receiving incentives and SMS reminders prior to the immunization due date increase the uptake of the measles vaccine? NI-ABAE will use this information to refine their program ahead of a large cluster RCT to measure the impact of the program on immunization coverage. This study was funded by GiveWell, a non-profit organization, that is dedicated to finding great giving opportunities and publishing details of their analysis to help donors decide where to give their donations.

## Methodology

### Study setting

The RCT was conducted in Nigeria between May 12^th^ and September 11, 2017, in conjunction with NI-ABAE. The intervention ran from 12^th^ May to July 12^th^ July, 2017, and outcome data was collected until the end of the study period. Participants were selected using NI-ABAE’s infant immunization records collected between October 24^th^, 2016 and April 25^th^ 2017. The trial was conducted in nine NI-ABAE’s pilot clinics across three states: Nasarawa (in the North Central region), Anambra (in South South), and Akwa Ibom (in South South).

This research was approved by the National Health Research Ethics Committee of Nigeria (NHREC/01/01/2007-07/08/2017) on August 7^th^, 2017, before any data was received by the researchers. Additionally, the Pre-Analysis Plan was registered in the 3ie’s RIDIE evaluation registry (RIDIE-STUDY-ID-5a394db3018d0). The trial protocol can be found on the RIDIE website. The delay in trial reregistration was because the study was originally simple A/B testing within NI-ABAE’s operational model and not intended for publication. The authors confirm that all ongoing and related trials for this drug/intervention are registered.

NI-ABAE considered several factors before choosing clinics for the pilot: clinics’ vaccination retention rates, volume, available supply and equipment needed for immunizations, available documentation, and immunization days. Retention is defined as the percentage of babies who complete their immunization schedule within nine months among those that receive the BCG immunizations. These clinics were used to pilot NI-ABAE’s operations and refine the components of the CCT program ahead of starting a large-scale, three state RCT of NI-ABAE’s program.

### Treatment assignment

Before this study was designed, NI-ABAE randomly allocated its pilot clinics to one of two models of its CCT program to explore which model yielded the highest uptake rate. In Model 1, caregivers received larger incentives than those in Model 2. The incentive amounts of these models determined the baseline incentive amounts in this study.

To allocate pilot clinics to the two models, the NI-ABAE did a stratified randomization based on region (North vs South) and state. There were two states per region, and three clinics per state; therefore the stratification could achieve balance at the region (but not the state) level. Initially, there were 12 clinics in total, however, three clinics in the Federal Capital Territory (FCT) were dropped from the study when NI-ABAE stopped its operations in those clinics due to regulatory issues. Since FCT had 2 clinics assigned to Model 1 and 1 clinic assigned to Model 2, dropping resulted in our sample having 1 more Model 2 clinic than Model 1 clinics (5 vs 4). It also meant that there were more Model 1 clinics in the South vs the North. We will come back to this issue when we discuss differences in results found between Model 1 and Model 2 clinics.

Within each clinic, eligible caregiver-child pairs were identified. Caregiver-child pairs were eligible for this study if the infant: a) was nine months or older, b) had received at least one previous CCT at an NI-ABAE clinic, c) had received their Penta-3 vaccine but had not yet received their measles vaccines, and d) the caregiver had provided a phone number (either a personal number or a number of someone who can reach them) during registration. Note that all the caregiver-child pairs in the study stood to receive only the measles incentives as NI-ABAE has a policy of paying the incentive for the most “valuable” immunizations if an infant receives multiple incentivized immunizations in one visit.

A total of 1088 caregiver-child pairs were selected from eligible pairs, stratified by clinic, and randomized to the treatment arms. This list included children’s whose measles immunization due dates fell within our study timeline. Using STATA 14 [16], we sorted caregiver-child pairs by measles immunization due date and then employed block randomization, with a block size of 8, to allocate the caregiver-child pairs to one of the four arms: 1) control (baseline amount of 2000 NGN or 3000 NGN), 2) baseline amount plus a reminder call, 3) baseline amount plus 1000 NGN and a reminder call, and 4) baseline amount plus 3000 NGN and a reminder call. This resulted in 96 caregiver-child pairs to each of the Model 1 arms and 176 pairs to each of the Model 2 arms (Table 2A).

**Table 2:** a. Treatment arms and number of participants. b. Summary of treatment arms (N = 1088).

	Description	Additional incentive amount (NGN)	Total incentive amount for Measles (NGN)	Reminder Call Made	Number of Caregivers			% of total sample
** **						**North**	**South**	
**Model 1 (2000 NGN)**	Baseline, no call	0	2000	No	16	80		8.8
	Baseline, call	0	2000	Yes	16	80		8.8
	Baseline + 1000 NGN + call	1000	3000	Yes	16	80		8.8
	Baseline + 3000 NGN + call	3000	5000	Yes	16	80		8.8
**Model 2 (3000 NGN)**	Baseline, no call	0	3000	No	82	94		16.1
	Baseline, call	0	3000	Yes	82	94		16.1
	Baseline + 1000 NGN + call	1000	4000	Yes	82	94		16.1
	Baseline + 3000 NGN + call	3000	6000	Yes	82	94		16.1
** **	**Description**	**Additional incentive amount (NGN)**	**Total incentive amount for Measles (NGN)**	**Reminder Call Made**	**Number of Caregivers**			**% of total sample**
** **						**North**	**South**	
**Model 1 (2000 NGN)**	Baseline, no call	0	2000	No	16	80		8.8
	Baseline, call	0	2000	Yes	16	80		8.8
	Baseline + 1000 NGN + call	1000	3000	Yes	16	80		8.8
	Baseline + 3000 NGN + call	3000	5000	Yes	16	80		8.8
**Model 2 (3000 NGN)**	Baseline, no call	0	3000	No	82	94		16.1
	Baseline, call	0	3000	Yes	82	94		16.1
	Baseline + 1000 NGN + call	1000	4000	Yes	82	94		16.1
	Baseline + 3000 NGN + call	3000	6000	Yes	82	94		16.1

While the number of available caregiver-child pairs was fixed by NI-ABAE’s operations, the study team conducted power calculations to help determine the number of treatment arms reasonable for the study, eventually settling on four arms per model. We assumed a baseline completion rate of 80% and standard 20% threshold for type-2 error, but a larger than normal 10% threshold for type-1 error and a since NI-ABAE was prepared to raise incentive sizes even if there was only weak evidence larger incentives would be beneficial. Given these assumptions, we are powered to detect a difference between arms of 4.5 percentage points in Model 1 and 3.3 percentage points in Model 2. The CONSORT [19] flow diagram is displayed in Fig 1.

**Fig 1:** CONSORT 2010 flow diagram.

### The implementation of the intervention

All participants randomized to receive a reminder call received the following text message a few days before the call: “*Please keep your phone on in the coming days*. *We will call you regarding your child [child’s name]*.” On the day of the call, the NI-ABAE’s team reminded caregivers of their child’s measles immunization date and the total amount of incentive they would receive once their child was vaccinated. If the caregiver could not be reached on the first attempt, the team made additional attempts at different times of the day on five different days across two weeks (up to 10 attempts were made per caregiver).

During the reminder calls, the team maintained a call log to ensure that a similar number of eligible caregivers for each experimental amount were called during the same week. This ensured that no group had a time advantage, i.e., receiving the call at the beginning of the week and, therefore, having more time to access their immunization than the other groups. These phone calls were conducted in the most commonly spoken local language of each state (Hausa for Nasarawa, Ibibio for Akwa Ibom, and Igbo for Anambra). Pidgin English was used as a backup language in all the states.

Two days after a successful reminder call, regardless of how many attempts were required, the caregivers received the following text message: “*Remember to vaccinate [child’s name] against Measles by [date like “end of month”] to protect it against disease and get [cash amount based on Group]*.” Once the caregiver had taken their child for immunization, they received their cash incentive after verification, and the NI-ABAE team recorded the immunization information. Note that all mothers, including those in the control group, received an automated reminder SMS prior to their scheduled due date.

### Data collection

Data was collected from two sources: NI-ABAE’s electronic administrative data and the phone log data. The administrative data comprising of the clinic name, the child’s unique ID, date of birth, and immunization date were recorded on the child health card. During cash disbursement, NI-ABAE collected data on the amount of money received from each immunization, the caregiver’s phone number and follow-up address, and transportation costs incurred to travel to the clinic. In cases where an NI-ABAE staff member was absent when children received their immunizations, we crosschecked the administrative data against immunization records. This only accounted for 3% of the days. However, if the child was immunized in another location, we did not record their information and they were considered unvaccinated for the purpose of this study. Since caregivers could only receive their cash payment by visiting their NI-ABAE clinic, we believe it is unlikely that many children were vaccinated in another location.

The phone log data was collected during the reminder calls to verify whether caregivers in the treatment groups received a call as planned. This data comprised of whether the caregiver was called, when they received the call, the treatment group they were in, and the child’s immunization status on the day of the call. If the primary caregiver could not be reached, the team called the alternative caregiver (if one was listed) for each call attempt.

### Outcomes

The primary outcome of interest was whether a child received the measles vaccine as recorded on the child’s health card. We defined a child as having completed the measles vaccine if she/he received the measles immunization at an NI-ABAE clinic any time before the end of the study period (September 12^th^ 2017). Note that the latest due date included in the study was July 30^th^, 2017. In addition to completion of measles vaccine, we also considered the average time between the child’s scheduled measles due date and actual immunization date. The child’s measles due date was constructed by adding nine months to the child’s date of birth as it appeared on her/his immunization card. We also analyzed the timeliness of other immunizations taken before measles using recorded dates of birth to generate due dates. Note, some birth dates may have been inaccurate if the caregiver did not receive the child’s health card on the actual date of birth.

### Data analysis

We first examined descriptive statistics for our overall sample and by model, including the average completion percentages for previous vaccines, number of days between the child’s immunization due date and the date of actual immunization, the number of days between the first phone call and the child’s measles due date, and one-way transportation costs to the clinic. All average proportions and mean values are presented with 95% confidence intervals. Additionally, Student’s T-tests with equal variance were used to assess differences in means and proportions between Model 1 and Model 2 households for all variables.

Secondly, to estimate impact of incentive size on the probability of a child completing her/his measles vaccine on time, we constructed unadjusted and adjusted linear probability models. In the adjusted models, the covariates included: receipt of BCG vaccine, receipt of PENTA (1–2) vaccine, receipt of pneumococcal vaccines, and time between the first call and measles vaccine due date. The Pre-Analysis Plan also included transportation costs as one of the covariates. However, since NI-ABAE only collected the transportation costs for caregivers who received the measles vaccines, we dropped it from our analysis. (This was due to a misunderstanding at the time of its writing, as the authors thought it would be collected for the entire evaluation sample.)

We tested the robustness of our findings by running our primary specifications using a probit model and constructing a linear probability model using a dummy variable for receiving a call, and a discrete variable for incentive size. Statistical significance was defined as a p-value < 0.05. All analyses were done using STATA 14 [16].

The analyses outlined in the Pre-Analysis Plan evaluated all treatment arms separately since NI-ABAE prioritized understanding what size incentive to offer for the measles vaccine. However, the regression coefficients were similar across all treatment arms, suggesting that the phone call, itself, may have increased measles coverage. Since this, too, was a policy-relevant question, we deviated from the Pre-Analysis Plan to pool the results and explore this new question.

We, therefore, considered a number of pooled models. The first model pooled all treatment arms (all arms that included a reminder call) and compared them to the control group (base incentive amount and no call). Under the assumption that increasing incentives does not increase immunization rates, this gives an estimate for the effect of providing a reminder call when incentives are already being offered. The second pooled model includes only caregivers who were not offered higher incentives; these caregivers were compared to those who did not receive a reminder call. This model estimated the effect of a reminder call without any additional assumptions but has lower power due to a restricted sample size. For both pooled models, we considered results separately for Model 1 and Model 2 clinics, as well as for the entire sample.

## Results

### Descriptive statistics

A total of 1088 caregivers from the nine pilot clinics were enrolled into the program—384 in Model 1 and 704 in Model 2 (Table 2B). There were 296 caregivers from Akwa Ibom (South South), 400 from Anambra (South East) and 392 from Nasarawa (North Central). In total, 696 (64%) caregivers were from the South and 392 (36%) from the North. However, the North-South split was not equal in the models; Model 1 had 17% (N = 64) of its caregivers from the North compared to 47% (N = 328) in Model 2.

When we looked at completion rates of the earlier scheduled vaccines; BCG, pentavalent, and pneumococcal vaccines, the overall sample had a 98.5% completion rate (Table 3). This completion rate is higher than other parts of Nigeria because the caregivers in the study were already enrolled onto the NI-ABAE program and had received the Penta-3 vaccine (two of the eligibility criterion) and their children had already received some or all of the initial vaccines. On average, these immunizations were completed within 23.5 days (95% CI: 14.6–32.6) to 51.3 (95% CI: 45.1–57.6) days from their due date, with Penta 3 recording the longest mean duration of 51 days. This indicates that many children received their immunizations later than expected. However, some infants (less than 5% for each vaccine) received immunizations prior to their due date possibly due to confusion on the part of the parents or clinic staff.

**Table 3:** Vaccine completion history and other descriptive characteristics.

			Model 1 (N = 384)				Model 2 (N = 704)		p-value^§^
	N		(%)	[95%CI]	N		(%)	[95% CI]	
BCG vaccine	378		98.4%	[97.2%, 99.7%]	674		95.7%	[94.2%, 97.2%]	0.02
Pentavalent-1	380		99.0%	[97.9%, 100.0%]	698		99.1%	[98.5%, 99.8%]	0.75
Pentavalent-2	381		99.2%	[98.3, 100.1%]	701		99.6%	[99.1%, 100.1%]	0.45
Pentavalent-3	384		100.0%		704		100.0%		
Pneumococcal-1	380		99.0%	[97.9%, 100.0%]	692		98.3%	[97.3%, 99.3%]	0.39
Pneumococcal-2	375		97.7%	[96.1%, 99.2%]	682		96.9%	[95.6%, 95.6%]	0.46
Pneumococcal-3	380		99.0%	[97.9%, 100.0%]	692		98.3%	[97.3%, 99.3%]	0.39
Measles vaccine	345		90.1%	[87.1%, 93.1%]	606		86.1%	[83.5%, 88.6%]	0.06
Call connected^b^	218		75.7%	[70.4%, 80.3%]	366		69.3%	[65.2%, 73.1%]	0.05
	Mean	Median [IQR]	Sd	[95% CI]	Mean	Median [IQR]	Sd	[95% CI]	
Days between BCG completion date and due date	24.6	8 [4,22]	116.32	[12.9, 36.4]	27.3	12 [5,31]	83.83	[21.0, 33.7]	0.67
Days between Penta (dose1) completion date and due date	20.8	5 [2,14.5]	116.88	[9.1, 32.6]	25.0	6 [2,16]	168.01	[12.5, 37.5]	0.67
Days between Penta (dose2) completion date and due date	27.8	10 [3,27]	117.81	[15.9, 39.6]	30.5	12 [4,29]	92.71	[23.6, 37.4]	0.68
Date between Penta (dose3) completion date and due date	49.5	30 [18,54]	123.43	[37.1, 61.9]	52.3	30 [21,54]	93.74	[45.3, 59.2]	0.68
Days between measles completion date and due date^a^	5.41	2 [0,6]	15.21	[3.81, 7.02]	4.90	2 [0,6]	16.28	[3.61, 6.20]	0.64
Days between first call and measles due date (days)^b^	3.96	0 [0,0]	14.52	[2.27, 5.65]	6.55	0 [0,1]	24.86	[4.44, 8.67]	0.10
One-way transportation cost (NGN)^c^	118.76	100 [50,150]	97.71	[108.08, 129.44]	108.57	100 [50,120]	98.31	[100.45, 116.69]	0.14

^§^ Difference in means and proportions using t-test between model 1 and model 2 households

^a^ Calculated for households who completed the measles vaccine. n = 952 (full model); n = 346 (Model 1); n = 606 (Model 2)

^b^ Calculated for households who received reminder calls. n = 816 (full sample); n = 288 (Model 1); n = 528 (Model 2)

^c^ Calculated for households who completed measles vaccine and reported average transport cost. n = 890 (full sample); n = 324 (Model 1); n = 566 (Model 2)

For the measles vaccine, there was an 87.5% completion rate in the overall sample [95% CI: 85.4% - 89.3%], and the average number of days between the completion date and due date was 5.09 days [95% CI: 4.08–6.10]. However, there was a slight variation between Model 1 and Model 2; Model 1 had a completion rate of 90.1% [95% CI: 87.1% - 93.1%], while Model 2 had a completion rate of 86.1% [95% CI: 83.5% - 88.6%], but this difference was not statistically significant (p-value = 0.06).

On call connectivity, 71.6% of the calls connected to those who were randomized to receive reminder calls in the full sample. However, this varied between Model 1 and Model 2. Call connection rates in Model 1 households (75.7%, 95% CI: 70.4%-80.3%) were 6 percentage points higher than Model 2 households (69.3%, 95% CI: 65.2%-73.1%). The p-value of this difference is 0.05). On average in the full sample, these calls were made about 5.6 days prior to the measles vaccine due date [95% CI: 4.15–7.13]. However, Model 1 households received their reminder calls 4.0 days prior to the due date [95% CI: 2.27–5.65] compared to Model 2 households where they received their calls 6.6 days before the due date [95% CI: 4.44–8.67]. This difference, however, was not statistically significant (p-value = 0.10).

### Effect of increased incentive amounts on completion rates

Reminder calls and increasing incentive sizes had heterogeneous effects (Table 4A). In the overall sample, there was no clear trend that increasing the incentive amount resulted in increased probability of completing the measles vaccine. However, when we look at the models separately, we see a significant effect in Model 1 households (Table 4B).

**Table 4:** a. Regression of total incentive amounts on measles coverage, full sample. b. Regression of incentives on measles coverage, by model.

	Unadjusted (N = 1088)			Adjusted* (N = 1088)		
** **	Coeff	[95% CI]	p-value	Coeff	[95% CI]	p-value
**Study arm**						
**Baseline incentive amount, no reminder call**	Ref (.838)			Ref (.878)		
**2000 NGN + call**	0.073	[-0.022, 0.168]	0.13	0.072	[-0.017, 0.161]	0.11
**3000 NGN + call**	0.023	[-0.052, 0.097]	0.55	0.026	[-0.045, 0.097]	0.48
**3000 NGN + call, (M1)**	0.083	[-0.010, 0.177]	0.08	0.077	[-0.011, 0.165]	0.09
**4000 NGN + call**	0.028	[-0.046, 0.102]	0.45	0.034	[-0.036, 0.104]	0.34
**5000 NGN + call**	0.115	[0.027, 0.202]	**<0.01**	0.115	[0.035, 0.195]	**<0.01**
**6000 NGN + call **	0.028	[-0.046, 0.102]	0.45	0.034	[-0.037, 0.104]	0.35
**BCG (tuberculosis) vaccine**				0.009	[-0.108, 0.127]	0.87
**Pentavalent vaccine, dose1**				0.01	[-0.199, 0.219]	0.93
**Pentavalent vaccine, dose2**				-0.144	[-0.301, 0.014]	0.07
**Pneumococcal vaccine, dose1**				0.026	[-0.209, 0.261]	0.83
**Pneumococcal vaccine, dose2**				-0.019	[-0.184, 0.146]	0.82
**Pneumococcal vaccine, dose3**				0.111	[-0.168, 0.391]	0.43
**Time between first call and measles due date (days)**				-0.005	[-0.010, -0.003]	**<0.01**
Baseline amount + no call	Ref (0.833)			Ref (0.841)		
Baseline amount + call only	0.073	[-0.023, 0.168]	0.13	0.023	[-0.052, 0.097]	0.55
1000 NGN + call	0.083	[-0.010, 0.177]	0.08	0.028	[-0.046, 0.102]	0.45
3000 NGN + call	0.115	[0.027, 0.202]	**<0.01**	0.028	[-0.046, 0.102]	0.45
Adjusted**						
Baseline amount + no call	Ref (0.790)			Ref (0.796)		
Baseline amount + call only	0.065	[-0.023, 0.153]	0.15	0.026	[-0.045, 0.097]	0.47
1000 NGN + call	0.064	[-0.023, 0.150]	0.15	0.033	[-0.038, 0.104]	0.36
3000 NGN + call	0.118	[0.039, 0.196]	**<0.01**	0.034	[-0.037, 0.104]	0.35
BCG (tuberculosis) vaccine	0.259	[-0.071, 0.588]	0.12	-0.049	[-0.158, 0.059]	0.37
Pentavalent vaccine, dose1	-0.103	[-0.189, -0.017]	**0.02**	0.069	[-0.251, 0.388]	0.67
Pentavalent vaccine, dose2	-0.314	[-0.500, -0.128]	**<0.01**	-0.102	[-0.325, 0.121]	0.37
Pneumococcal vaccine, dose1	-0.037	[-0.138, 0.064]	0.427	0.047	[-0.249 0.343]	0.76
Pneumococcal vaccine, dose2	0.076	[-0.184, 0.335]	0.566	-0.014	[-0.232 0.205]	0.9
Pneumococcal vaccine, dose3	0.205	[-0.212, 0.621]	0.335	0.117	[-0.223 0.458]	0.5
Time between first call and measles due date (days)	-0.008	[-0.010, -0.006]	**<0.01**	-0.004	[-0.006, -0.002]	**<0.01**

*In the adjusted models, the covariates included: BCG, PENTA (1–3), pneumococcal vaccines, and the time between the first call and the measles vaccines. Pentavalent vaccine dose 3 is excluded from results because of collinearity as the results are 100% (all study participants had received this vaccine).

**In the adjusted models, the covariates included: BCG, PENTA (1–3), pneumococcal vaccines, and the time between the first call and the measles vaccines. Pentavalent vaccine dose 3 is excluded from results because of collinearity as the results are 100% (all study participants had received this vaccine). Note that the other vaccine co-variates are also highly collinear as 98.5% of the sample completed all previous vaccines, but these controls were pre-specified as we anticipated lower completion rates. Removing the vaccine controls doesn’t affect the model 2 results, it does make the coefficient on the 1000 NGN + call and call only arms slightly higher:0.075 ([95% CI: 0.011–0.162] p-value = 0.09) and 0.079 ([95% CI: -0.009–0.167] p-value0 = .08) respectively.

In Model 1 households, an additional 1000 NGN and 3000 NGN resulted in an adjusted 6.4 percentage point (95% CI: -2.3–15, p-value = 0.15) and 11.8 percentage point (95% CI: 3.9–19.6, p-value<0.01) increase in the probability of completing the measles vaccines, respectively. These increases correspond to an 8% and 15% increase relative to the 79% adjusted coverage in the no call group. Only the 3000 NGN increase was significant. On the other hand, in Model 2 households, increasing the incentive by 1000 NGN and 3000 NGN increased the adjusted probability by 3.3 (95% CI: -3.8–10.4, p-value = 0.36) and 3.4 (95% CI: -3.7–10.4, p-value = 0.35) percentage points respectively or a 4% relative increase. However, these increases were not statistically significant.

### Effects of reminder calls on completion rates

Adding reminder calls to incentives increased the probability of completing the measles vaccine; when pooling all treatment arms (including those which included an increased incentive) and adjusting for covariates caregivers who received reminder calls were 5.1 percentage points more likely to get their children vaccinated in the full sample (95% CI: 0.50–9.8, p-value = 0.03) compared to those who did not receive a reminder call (Table 5). This effect was largely driven by Model 1 households; households that received incentives plus reminder calls were 8.3 percentage points more likely to complete measles vaccines (95% CI: 0.9–15.6 percentage points, p-value = 0.03) than Model 1 households who did not receive any reminder calls. In Model 2, incentives plus reminder calls increased the probability of completing the measles vaccine by 3.1 percentage points (95% CI: -2.8–9.0 percentage points) compared to those who did not receive a call. This increase, however, was not statistically significant (p-value = 0.30).

**Table 5:** Effect of reminder calls on uptake of measles vaccine (pooled results).

	Model 1 households (N = 384)			Model 2 households (N = 704)			Full sample (N = 1088)		
Unadjusted									
	Coef	[95% CI]	p-value	Coef	[95% CI]	p-value	Coef	[95% CI]	p-value
Study arm									
No reminder call	Ref (0.833)			Ref (0.841)			Ref (0.838)		
Received a reminder call	0.090	[0.009, 0.172]	**0.03**	0.027	[-0.035, 0.088]	0.40	0.049	[0.004, 0.094]	**0.03**
Adjusted*									
No reminder call	Ref (0.797)			Ref (0.800)			Ref (0.864)		
Received a reminder call	0.083	[0.009, 0.156]	**0.03**	0.031	[-0.028, 0.090]	0.30	0.051	[0.005, 0.098]	**0.03**
BCG (tuberculosis) vaccine	0.24	[-0.091, 0.570]	0.16	-0.050	[-0.156, 0.056]	0.35	0.007	[-0.110, 0.123]	0.91
Pentavalent vaccine, dose1	-0.080	[-0.157, -0.003]	**0.04**	0.0672	[-0.251, 0.386]	0.68	0.010	[-0.195, 0.215]	0.92
Pentavalent vaccine, dose2	-0.295	[-0.473, -0.117]	**<0.01**	-0.102	[-0.325, 0.121]	0.37	-0.134	[-0.289, 0.022]	0.09
Pneumococcal vaccine, dose1	-0.050	[-0.136, 0.035]	0.25	0.046	[-0.249, 0.341]	0.76	0.023	[-0.211, 0.257]	0.85
Pneumococcal vaccine, dose2	0.068	[-0.184, 0.321]	0.60	-0.013	[-0.231, 0.205]	0.91	-0.018	[-0.182, 0.145]	0.83
Pneumococcal vaccine, dose3	0.195	[-0.228, 0.617]	0.37	0.117	[-0.223, 0.456]	0.50	0.113	[-0.168, 0.394]	0.43
Time between first call and measles due date (days)	-0.008	[-0.010, -0.006]	**<0.01**	-0.004	[-0.006, -0.002]	**<0.01**	-0.005	[-0.007, -0.003]	**<0.01**

*In the adjusted models, the covariates included: BCG, PENTA (1–3), pneumococcal vaccines, and the time between the first call and the measles vaccines. Pentavalent vaccine dose 3 is excluded from results because of collinearity as all study participants had to receive this vaccine to be eligible for the study. Removing the vaccine controls yields results nearly identical to the unadjusted results.

In the absence of added incentives (baseline incentive amount only), the reminder call increased the probability of measles completion by an adjusted 4.2 percentage points (95% CI: -1.40–9.71 percentage points) compared to those who did not receive a reminder call in the full sample (Table 6). This increase, however, was not statistically significant (p-value = 0.14). When we looked at the models separately, reminder calls in Model 1 increased the adjusted probability of completing measles vaccines by 5.8 percentage points (95% CI: -3.1–14.8 percentage points, p-value = 0.20), whilst in Model 2, the reminder call increased the adjusted probability of measles completion by 2.2 percentage points (95% CI: -4.90–9.3 percentage points, p-value = 0.54). Neither of these results by individual model were statistically significant.

**Table 6:** Effect of reminder calls on uptake of measles vaccine, among households with baseline incentive amounts only.

	Model 1 households (N = 192)			Model 2 households (N = 352)			Full sample (N = 544)		
Unadjusted									
	Coef	[95% CI]	p-value	Coef	[95% CI]	p-value	Coef	[95% CI]	p-value
Study arm									
Baseline incentive amount, no reminder call	Ref (0.833)			Ref (0.841)			Ref (0.838)		
Baseline incentive amount, with reminder call	0.073	[-0.023, 0.169]	0.14	0.023	[-0.052, 0.097]	0.55	0.040	[-0.018, 0.099]	0.18
Adjusted*									
Baseline incentive amount, no reminder call	Ref			Ref			Ref		
Baseline incentive amount, with reminder call	0.058	[-0.031, 0.148]	0.20	0.022	[-0.049, - 0.093]	0.54	0.042	[-0.014, 0.097]	0.14
BCG (tuberculosis) vaccine	0.359	[-0.379, 1.098]	0.34	-0.146	[-0.251, -0.041]	**<0.01**	-0.073	[-0.255, 0.108]	0.43
Pentavalent vaccine, dose1	-0.073	[-0.134, -0.012]	**0.02**	0.472	[-0.150, 1.094]	0.14	0.153	[-0.342, 0.647]	0.55
Pentavalent vaccine, dose2	-0.193	[-0.357, -0.029]	**0.02**	0.155	[-0.113, 0.423]	0.26	-0.136	[-0.402, 0.129]	0.31
Pneumococcal vaccine, dose1	-0.303	[-1.081, 0.476]	0.44	0.458	[-0.013, 0.929]	0.06	0.355	[-0.068, 0.777]	0.36
Pneumococcal vaccine, dose2	-0.046	[-0.146, 0.054]	0.36	-0.244	[-0.503, 0.015]	0.06	-0.213	[-0.370, -0.055]	**<0.01**
Pneumococcal vaccine, dose3	0.319	[-0.207, 0.844]	0.23	0.0346	[-0.260, 0.329]	0.82	0.124	[-0.157, 0.405]	0.39
Time between first call and measles due date	-0.008	[-0.011, -0.005]	**<0.01**	-0.005	[-0.007, -0.003]	**<0.01**	-0.006	[-0.008–0.004]	**<0.01**

a*In the adjusted models, the covariates included: BCG, PENTA (1–3), pneumococcal vaccines, and the time between the first call and the measles vaccines. Pentavalent vaccine dose 3 is excluded from results because of collinearity as all study participants had to recieve this vaccine to be eligible. Removing the other vaccine controls makes the model 1 pooled specification marginally significant with a coefficient of 0.079 ([95% CI: -0.010-.168] p-value = 0.08)

## Discussion

This study demonstrates that a combination of incentives and reminder calls can modestly increase the uptake of the measles vaccine. These findings are similar to studies conducted in India and Kenya which found that increasing incentives [9,13] and reminding caregivers about immunization due dates increases immunizations rates. [2,13,17]

However, higher incentives only led to increased immunizations in Model 1 households, suggesting that the incentive size may not be as important as simply receiving a reminder call for caregivers already enrolled in the program. [9,14] These findings are similar to Banerjee et al. (2010) and Filmer and Schady’s studies (2009), which revealed that the highest incentive did not result in the highest increases in immunization rates or school enrollment. These authors posit that there is a law of diminishing returns as incentive size increases and that the larger incentive is not as attractive as a smaller incentive.

The differing results between model 1 and model 2 clinics could have many possible explanations. In terms of the limited available observables, model 1 and model 2 are similar. There was no statistically significant difference in estimated transportation costs between model 1 and model 2 caregivers. Similarly, there are no statistically significant differences in measles due dates which means the model 1 population didn’t contain significantly more caregivers who were months past their due date at the time of the first reminder call.

Differences in the geographic split in the number of caregivers in the models may also have contributed to the difference in uptake rates. Due to the aforementioned regional imbalance, Model 2 had twice the percentage of caregivers from the northern state of Nasarawa than Model 1. (Nasarawa was the only Northern state included in the study.) As highlighted in the introduction, Nasarawa has much lower immunization rates than the South, and therefore the factors that prevent caregivers in the North from immunizing their children on time may have played a role in these results. Notably, in the 2018 DHS study 9% of women in Nasarawa said they have the final say in their own health care as compared to 81% in Akwa Ibom and 98% in Anambra [18]. Other notable differences between Nasarawa and the southern states include Islam vs Christianity as the dominant religion, substantially lower wealth and female literacy (60% in Nasarawa vs 80 in Akwa Ibom and 87% in Amnambra in DHS 2018) [18]. However, we do not see different treatment effects in the North vs South, which complicates reliance on any regional explanation for the different results between models.

Overall, our observable data does not give a clear explanation for why the program was more successful in Model 1 clinics than in Model 2 clinics. Given the small number of clinics, there are likely unobserved idiosyncratic differences between the clinics in the two models that are driving the different behaviors in the different models. For instance, this could be population density or the existence of alternative vaccination providers.

### Strengths of this study

This study used randomization methodology to allocate clinics to the two models and caregivers to the treatment arms, thus providing an unbiased estimate of the treatment arms’ impacts. Secondly, this study used a combination of texts and calls to communicate about future immunization, where previous studies have used only one, mainly text messages. This increased our chance of communication with the caregivers, particularly those with lower literacy levels.

### Limitations of this study

The study’s eligibility criteria and study area make it difficult to generalize these findings to the complete Nigerian context and to areas that need to increase immunization rates the most, i.e., areas with low immunization rates like North Nigeria tend to be areas with low mobile phone penetration and/or low network connectivity. First, the study selected caregivers who were already enrolled onto the NI-ABAE program and had access to a mobile phone, and whose children had already received previous immunizations. These characteristics are specific to this population and may not be representative of the general population. In this context, our control group (caregivers enrolled in the CCT program) had immunization rates of around 84%. The control group also received reminder SMS messages, which may have increased immunization rates. Therefore, the setting may not provide as much information about the effect of incentives as one with a lower baseline immunization rate.

Finally, this study did not explore factors related to why caregivers do or do not immunize their children. Therefore, we do not understand how and why Model 1 and Model 2 caregivers may have differed from each other, nor the barriers that prevented caregivers from taking their children for immunization.

### Policy implications

This study demonstrates that incentives and reminders can modestly increasing the uptake of the measles vaccine. In addition, the study suggests that in certain contexts calling reminders can enhance the impact of an incentive program. However, the program also shows that there is substantial regional heterogeneity in response to both incentives and calls. While one possible conclusion is that larger incentives and phone reminders are more likely to work in higher income and higher baseline coverage settings, the study is not designed to evaluate this claim. Rather, policymakers could consider experimenting with a similar low-cost calling study as part of the design of other cash transfer programs to identify whether adding reminder phone calls could increase the impact of the program.

Optimizing transfer amounts can also result in substantial cost savings. For example, the marginal cost of this study for NI-ABAE was only three call center operators working part-time for three months but reducing the incentive by 1000 NGN for the 10000 infants saves NI-ABAE nearly 28,000 USD (Based on 360 NGN = 1 USD). Implementers need to determine the optimal incentive amount that would yield the highest uptake at a minimum cost. Other implementers should note, that this experiment was only possible because NI-ABAE kept routine program data in an easy to analyze electronic format. This study serves as a case study of the types of analysis that are possible when implementers invest in robust monitoring.

In areas with low mobile phone penetration and poor network coverage, NI-ABAE or other implementers could still experiment with randomizing different outreach strategies using a robust monitoring system to collect outcome data. For example, in the resource constrained North West Nigeria, NI-ABAE utilizes town criers and local religious and community leaders to announce immunization days. By randomizing the hamlets that receive these services, NI-ABAE could assess the impact of these outreach efforts empirically.

Subsequent to this study NI-ABAE shifted operations to Jigawa, Katsina, and Zamfara in Nigeria’s North West. Given the low cell-phone penetration rates in these states New Incentives has focused on in-person outreach efforts and discontinued all phone reminders including SMS. The authors’ research has shifted to studying the effectiveness of NI-ABAE’s modified program in the North West where they intend to scale. The evaluation is a cluster randomized controlled trial based on in-person coverage surveys within clinic catchments. These surveys will explore barriers to immunization for caregivers in North West Nigeria in some depth.

Future research on phone reminders should examine the impact of calling reminders for other incentive programs or for immunization programs without cash incentives. Additionally, they could explore the mechanism through which phone-based reminders influence immunization coverage. This would give us a better understanding of how implementers can refine their programs to reach the maximum level of impact.

## Supporting information

S1 File Anonymized data. (CSV)

S1 Checklist CONSORT 2010 checklist of information to include when reporting a randomised trial*. (DOCX)

S1 Data (PDF)
